# *Artemisia* Extracts and Artemisinin-Based Antimalarials for COVID-19 Management: Could These Be Effective Antivirals for COVID-19 Treatment? †

**DOI:** 10.3390/molecules27123828

**Published:** 2022-06-14

**Authors:** Pawan K. Agrawal, Chandan Agrawal, Gerald Blunden

**Affiliations:** 1 Natural Product Inc., 7963 Anderson Park Lane, Westerville, OH 43081, USA; editorial@naturalproduct.us; 2 School of Pharmacy and Biomedical Science, University of Portsmouth, Portsmouth PO1 2DT, UK; gblunden10@gmail.com

**Keywords:** *Artemisia*, artemisinins, antiviral, drug repurposing, COVID-19

## Abstract

As the world desperately searches for ways to treat the coronavirus disease 2019 (COVID-19) pandemic, a growing number of people are turning to herbal remedies. The *Artemisia* species, such as *A. annua* and *A. afra*, in particular, exhibit positive effects against severe acute respiratory syndrome coronavirus-2 (SARS-CoV-2) infection and COVID-19 related symptoms. *A. annua* is a source of artemisinin, which is active against malaria, and also exhibits potential for other diseases. This has increased interest in artemisinin’s potential for drug repurposing. Artemisinin-based combination therapies, so-called ACTs, have already been recognized as first-line treatments against malaria. *Artemisia* extract, as well as ACTs, have demonstrated inhibition of SARS-CoV-2. Artemisinin and its derivatives have also shown anti-inflammatory effects, including inhibition of interleukin-6 (IL-6) that plays a key role in the development of severe COVID-19. There is now sufficient evidence in the literature to suggest the effectiveness of *Artemisia*, its constituents and/or artemisinin derivatives, to fight against the SARS-CoV-2 infection by inhibiting its invasion, and replication, as well as reducing oxidative stress and inflammation, and mitigating lung damage.

## 1. Introduction

One of the biggest breakthroughs in fighting the COVID-19 pandemic has been the development of vaccines that provide the best strategies to prevent infection against COVID-19. Several vaccines have been approved by the U.S. Food and Drug Administration (FDA). These have been shown to be highly effective and are available to the public for emergency use authorization (EUA) and for protection against COVID-19 [1]. These vaccines are safe and effective, since, in the rare instances of breakthrough infections (where a person has been vaccinated against COVID-19), patients are significantly less likely to become hospitalized. While vaccines prevent disease occurrence, infected individuals still need other treatment options.

Viral infection happens when a virus inserts its genetic code into a host cell, forcing it to replicate, produce more viral genomic material, and then leads to the death of the host cell. During a viral infection, this process can happen at enormous rates, which leads to viral fever affecting primarily the respiratory tract system, harmful inflammation, and excessive aberrant immunological responses as the body’s immune system tries to seek out and destroy viral material and, at a later stage, it can lead to potentially deadly complications [2,3,4]. By preventing virus entry and/or its replication or clearing of cells into which the virus has already entered, effective treatments with antivirals can help to slow the spread of a person’s infection, potentially reducing the length and severity of symptoms. Thus, safe and effective antivirals responsible for restricting viral entry and/or disruption of the replication process are crucial to the pandemic response [5,6,7,8,9,10,11,12,13].

Despite vaccine developments, COVID-19 treatment still remains largely supportive with an urgent need to identify effective anticoronavirals. An attractive approach is repurposing drugs already licensed for other diseases. In this respect, several studies have been undertaken to test whether antimalarial drugs could treat COVID-19. Teas of *Artemisia annua* L. plants have been employed to treat malaria [14,15,16] in many African countries. Scientists are currently testing *A. annua*’s potential against SARS-CoV-2, as it provides a basis for a large variety of derivatives used as antimalarial drugs, collectively called “artemisinins”. In the present review, we summarize the antiviral significance of two *Artemisia* species, namely *A. annua* and *A. afra* Jacq. ex Willd., as well as artemisinins.

## 2. Traditional Use and Bioactive Compounds of *Artemisia*

*Artemisia annua* (“sweet wormwood”, “qinghao”), a member of the Asteraceae family, has been traditionally used safely over the centuries to treat a variety of fevers, and notably, ‘‘intermittent fevers” and chills-related conditions, including respiratory tract infections [17,18,19,20]. One of the most bioactive compounds identified is a sesquiterpenoid lactone, artemisinin (**1**), which contains an unusual 1,2,4-trioxane moiety with an endoperoxide group. This compound has been identified as an active ingredient to treat malaria infections. This unusual endoperoxide bridge is the key active site for its drug mechanism of action and provides a structural chemical base for the synthesizing of a large variety of compounds, such as dihydroartemisinin (**2**), β-artemether (**3**), and artesunate (**4**) (Figure 1), exhibiting greater potency, improved water solubility, and improved pharmacological properties [21]. These artemisinin derivatives are the components of artemisinin-based combination therapies (ACTs), which have been approved as front-line drugs for treating *Plasmodium falciparum* malaria [22,23,24]. They also show additional pharmacological benefits such as anticancer, anti-inflammatory, and immunomodulatory properties [25,26,27,28,29,30,31,32,33]. In addition, *A. annua* has been extensively investigated and more than 600 chemical constituents have been identified [18,19,20,21,22,23,24,25,26,27,28,29,30,31,32,33,34,35,36,37,38,39,40].

The artemisinin derivatives artesunate and artemether are the key ingredients of the WHO-recommended antimalaria combination therapies [41,42]. *A. annua* extracts and their constituents are active against several viruses, including SARS-CoV [43,44,45], suggesting the usefulness of artemisinin’s potential for drug repurposing.

## 3. Anti-Viral and Immune-Stimulatory Potential of *Artemisia*

In 2002, Lin et al., reported the use of *A. annua* against SARS coronavirus [46]. Interestingly, in a Vero cell-based, 3-(4,5-dimethylthiazol-2-yl-)-5-(3-carboxymethoxyphenyl)-2-(4-sulfophenyl)-2H-tetrazolium inner salt (MTS) assay for virus-induced cytopathic effect (CPE) screening analysis of medicinal plant extracts with antiviral potentials against SAR-CoV viral strain BJ001, *A. annua*, alongside three other plants, demonstrated a substantial inhibitory effect [46]. The ethanolic extract of whole plants of *A. annua* showed potent antiviral activities with 50% effective concentration (EC_50_) values of 34.5 (±2.6) and 39.2 (±4.1) μg/mL against the SARS-CoV-1 viral strains BJ-001 and BJ-006, respectively, with a CC_50_ value of 1053.0 ± 92.8 μg/mL in a cytotoxicity assay [47]. Ethnopharmacological studies of *Artemisia* and its constituents have also revolved around their retroviral properties [43,47,48,49,50], capacity to minimize the replication of herpes viruses [43,51,52,53,54], and activity against bovine viral diarrhoea, Epstein–Barr virus, hepatitis B virus, and hepatitis C virus [55,56,57,58,59,60,61,62]. Interestingly, derivatization enhanced the antiviral activity of artemisinin as its derivatives, i.e., artesunate, artemether, and arteether, including dimer and trimer molecules, exhibited potent antiviral activities [62]. For example, artesunate effectively inhibits human cytomegalovirus (HCMV), human herpes simplex virus (HSV), hepatitis B virus (HBV), hepatitis C virus (HCV), human immunodeficiency virus (HIV), and polyomavirus BK [43,63,64]. Dihydroartemisinin has also shown inhibitory effects on HCMV and Zika virus [65,66], whereas artemisone, alone and in combination with other anti-HCMV agents, has been proven to be a potent HCMV inhibitor [67,68]. Artemisinin inhibited the replication of hepatitis C replicon, a single-stranded RNA virus, similar to SARS-CoV-2 [69]. A recent review by Efferth provided up-to-date information about the inhibition of viruses by artemisinin-type compounds [62].

The presence of flavonoids, such as quercetin and rutin, in *Artemisia* species can be associated with inhibition of activity of the main protease (M^pro^), also known as chymotrypsin-like protease (CL^pro^), an enzyme intrinsic for replication of SARS-CoV-2 [70,71,72,73,74]. The presence of various bioactive components in *A. annua* seems to be responsible for its adoption as a therapeutic option against coronavirus infection. *Artemisia* also contains a high concentration of zinc, which has been reported to have an immunomodulation effect on the host response [75]. It should also be noted that the antioxidant ability of *Artemisia* has been shown to enhance immune defence [30,76]. The tea infusion of *A. annua* has shown potent anti-HIV activity, with a half maximal inhibitory concentration (IC_50_) of 2.0–14.8 µg/mL in vitro. The tea infusion was lacking in artemisinin, suggesting that the anti-HIV activity may be associated with other compounds [50].

Thus, the antiviral and antimalarial significance of *A. annua* and artemisinin derivatives have led to exploring their diverse pharmaceutical potentials [76,77]. Furthermore, earlier pharmacokinetic, pharmacodynamic, and cytotoxicity studies have identified additional factors that made them potential candidates for drug repurposing [78,79,80,81]. Thus, the COVID-19 pandemic outbreak has attracted attention on the efficacy and repurposing of the multifunctional properties of *Artemisia* and artemisinin-derived products as promising therapeutic drugs for the possible treatment of SARS-COV-2 [81,82].

Some antimalarial and/or antiviral agents, such as chloroquine (CQ), hydroxychloroquine (HCQ), and redmesivir, have been repurposed for their possible use against COVID-19 [83]. However, these may have caused cardiotoxicity concerns, as well as other after-administration side effects [84]. However, notably, artemisinin has been reported to possess a better and lower toxicity profile [85].

## 4. *Artemisia* Extracts and COVID-19

In response to the pandemic, in April 2020, a herbal tea or decoction based on *Artemisia*, developed by the Malagasy Institute for Applied Research (IMRA), and branded as “COVID-Organics”, was launched as a cure for COVID-19. It contains 62% *Artemisia annua* and a mixture, in confidential proportions, of Malagasy medicinal plants used in the composition of traditional remedies, such as antiseptics and bronchial fluidizers. President Rajoelina of Madagascar said that trials conducted on the COVID-Organics drink showed its effectiveness against the disease [86]. However, the use of a tonic containing unknown quantities of artemisinin and other constituents, over a large population, certainly raises fears of malarial parasites developing resistance. Moreover, its widespread unregulated usage as remedies for malaria, such as in tea, could result in reduced access to effective medicines and possible resistance of *P. falciparum* to artemisinin-based combination therapies (ACTs) [87,88,89]. Since May 2020, IMRA has been preparing an injectable form of *Artemisia*-derived products for patients in respiratory distress. In a recent study by Nie et al., it was shown that several *Artemisia* extracts, as well as Covid-Organics, at concentrations that did not affect cell viability, inhibited SARS-CoV-2 and feline coronavirus (FCoV) infection [90].

In a study related to the efficacy of *A. annua* extracts in high-throughput antiviral in vitro assays in VeroE6 cells, Gilmore et al., found that the leaves, after being extracted with either pure ethanol or distilled water, showed antiviral activity and the activity increased considerably when the ethanol extract was combined with coffee [91]. Extracts were added to VeroE6 cells either 1.5 h prior to infection (pretreatment (pt)] or 1 h post infection (treatment (t)), followed by a two-day incubation of the virus with extracts. The EC_50_ values were 173 µg/mL (pt) and 142 µg/mL (t) for the ethanolic extract; 390 µg/mL (pt) and 260 µg/mL (t) for the aqueous extract; and 176 µg/mL (pt) and 128 µg/mL (t) for the ethanolic extract and coffee, respectively [91]. With all extracts, almost complete virus inhibition was achieved at high concentrations: Cell viability assays revealed median cytotoxic concentrations (CC_50_) of 1044 µg/mL (*A. annua* ethanolic extract), 632 µg/mL (*A. annua* + coffee ethanolic extract), and 2721 µg/mL (*A. annua* aqueous extract). Selectivity indexes (SI), determined by dividing CC_50_ by EC_50_, revealed similar results. For the *A. annua* ethanolic extract the SIs were 6 (pt) and 7 (t), for the *A. annua* + coffee ethanolic extract 3 (pt) and 5 (t), and for the *A. annua* aqueous extract 7 (pt) and 10 (t), respectively [92]. The use of dried *A. annua* leaves has also been suggested as a potential therapeutic and inexpensive option for treating SARS-CoV-2 infection [92].

Recently, hot water extract obtained from dried leaves of *A. annua*, obtained from four different parts of the world, was tested against SARS-CoV-2, and two variants, B1.1.7 and B1.351, showed IC_50_ values corresponding to <12 μM artemisinin [93,94,95]. It was also noticed that the antiviral effect of the extracts decreased in inverse correlation with the artemisinin content. The failure of the IC_50_ to decrease as the concentration of artemisinin and/or flavonoids increased, indicated that these were not the only active factors, but may, in fact, be antagonists of the bioactive component. The plant possesses compounds that inhibit inflammation and the formation of scar-like tissues known as fibrosis, which also affect patients with COVID-19, but this warrants further investigation [93,94,95].

In South Africa, teas of *Artemisia afra* were used without in vitro or clinical data [96]. *A. afra*, in contrast to *A. annua*, does not contain artemisinin. Due to fears that artemisinin combination therapies against malaria may become ineffective if artemisinin-based treatments are used against COVID-19 [97], the WHO recently called for investigations into the efficacy of plant-based traditional medicines [98]. Human clinical trials will be required to answer the question whether the traditional medicines may indeed have an effect in either preventing or treating COVID-19 infections.

A study by Zhou et al. [99] related to the in vitro efficacy of *A. annua* ethanolic and aqueous extracts, artemisinin, artesunate, and artemether against SARS-CoV-2 spike glycoprotein revealed that treatment with extracts and compounds inhibited SARS-CoV-2 infection of VeroE6 cells, human hepatoma Huh7.5 cells, and human lung cancer A549-hACE2 cells. In treatment assays, the range of 50% effective concentrations (EC_50_) ranged between 83 and 260 µg/mL for *A. annua* extracts [99].

The aqueous fraction of *A. annua*, after the extraction of artemisinin, has been shown to regulate the expression of proinflammatory cytokines, matrix metalloproteinases, and NF-κB; to promote cell cycle arrest; to drive reactive oxygen species production; and to induce Bak or Bax-apoptosis [17]. It has also been reported that among the three different ethanol extracts (50%, 70%, and 95%), only the 70% and 95% extracts showed any positive antiviral activity, and the 70% extract was considered to be optimum for further investigation, as the 95% ethanol extract could be associated with cellular toxicity [100].

In a recent study, hot-water extracts of *A. annua* were found to be active against SARS-CoV-2 and its alpha, beta, gamma, delta, and kappa variants. The *A. annua* cultivar with the lowest artemisinin content had the lowest (most effective) IC_50_ against gamma, delta, and kappa variants, thus, demonstrating the potential of the extracts as treatments against this virus [101]. However, clinical studies are required to further evaluate the utility of these teas/drinks/extracts for COVID-19 prevention.

## 5. *Artemisia* Supplement and Formulation

The Max Planck Institute of Colloids and Interfaces (Germany) is collaborating with a company in the USA, ArtemiLife Inc., to explore the effect of *A. annua* plant extract and artemisinin derivatives against SARS-CoV-2 [102]. ArtemiLife is also marketing *A. annua* herbal tea and coffee directly to consumers, but is careful to note that its tea and coffee are “not intended to diagnose, treat, cure or prevent any disease” and cautions that common side effects may include hearing loss and liver problems. However, it also claims that drinking two servings per day will help consumers “maintain an active shield,” thus, “protecting well-being.” The firm’s coffee contains 0.4 g *A. annua* per serving, and its tea containes 0.23 g. The dried leaves of *A. annua* usually contain around 1% artemisinin, therefore, consuming the drinks would offer much lower doses than typical ACTs [103].

The product, ARTIVeda/PulmoHeal, delivered in a gelatin capsule, is an Ayurvedic drug against COVID-19. The drug is a formulated extract of *Artemisia* for oral delivery of artemisinin for growth factor-β (TGF-β) inhibition. It targets COVID-19 by suppressing both viral replication and clinical symptoms, i.e., both viral and immune driven pathologies (ARDS and cytokine storm) that arise from viral infection. With treatment, viral replication is suppressed, IFNβ is induced, and innate and adaptive immune responses are suppressed. The clinical studies on patients with mild and moderate COVID-19 have suggested that administration of artemisinin 500 mg capsules once daily for 5 days may lead to a faster recovery [103].

In a controlled Phase II trial, patients with COVID-19 received ArtemiC, a medical spray (containing artemisinin, curcumin, frankincense resin from the *Boswellia sacra* tree, and vitamin C, in a nanoparticular formulation for spray administration), in addition to standard care; improvement in the patients’ condition was recorded [104].

## 6. Artemisinin and *Artemisinins*’ Potential in Management of COVID-19

In vitro efficacy of artemisinin-based treatments for combating SARS-CoV-2 has indicated that treatment with artesunate, artemether, *A. annua* extracts, and artemisinin hindered virus infections of human lung cancer A549-hACE2 cells, VeroE6 cells, and human hepatoma Huh7.5 cells. Among these four treatments, artesunate showed the strongest anti-SARS-CoV-2 activity (7–12 µg/mL), followed by artemether (53–98 µg/mL), *A. annua* extracts (83–260 µg/mL) and artemisinin (151 to at least 208 µg/mL). Collectively, time-of-addition experiments in A549-hACE2 cells displayed that artesunate attacked the virus at the post-entry level [103]. Dried-leaf, hot-water extracts of *A. annua* cultivars (SAM, BUR, A3, and MED) revealed in vitro anti-SARS-CoV-2 activity against alpha, beta, gamma, delta, and kappa variants of the virus. All cultivars, in addition to being potent in combating the original wild type WA1, also showed effective potential against the mentioned variants. The IC_90_ and IC_50_ values, according to measured artemisinin content, ranged from 1.4–25.0 µM and 0.3 to 8.4 µM, respectively. In addition, the IC_90_ and IC_50_ values, according to dried leaf weight, ranged from 59.5 to 160.6 µg DW and 11.0 to 67.7 µg DW, respectively [105].

It has also been reported that *A. annua* stimulated adaptive immunity by generating CD8 and CD4 lymphocytes responsible for the production of antibodies targeting SARS-CoV-2 and downregulating the production of proinflammatory cytokines [106]. Cytokine storms led to functionally exhausted CD8 and CD4 lymphocytes, which ultimately caused severe respiratory failure [107]. Interestingly, artemisinin and its derivatives also regulate multiple immune cells, including macrophages, monocytes, dendritic cells, and T cells to inhibit proinflammatory cytokine release and cytokine storm outbreak [108]. More clinical studies need to be conducted to provide further therapeutic protocols to substantiate the safety and efficacy of *Artemisia* either in monotherapeutic form or as combination therapies with existing drugs [109,110].

While extracts from *Artemisia* plants have shown efficacy in small-scale clinical trials, these have not clarified whether a specific chemical constituent is responsible or whether the effect is due to a synergistic antiviral effect of several compounds [109]. A recent study suggested that the antiviral and immunomodulation effects of *Artemisia* extracts may not only be due to artemisinin, but also to other potentially identified and/or unidentified bioactive compounds [20]. To address the efficiency and potential side effects of the extracts, detailed knowledge about the molecular mode of action of individual bioactive constituents is needed [17].

## 7. Artemisinin-Based Combination Therapies (ACTs)

The World Health Organization (WHO) has recommended the use of artemisinin-based combination therapies (ACTs) in the treatment of malaria (artemether-lumefantrine, artesunate-amodiaquine, dihydroartemisinin-piperaquine, and artesunate-mefloquine). Amodiaquine and mefloquine, two quinoline ACT partners, were active in vitro at micromolar concentrations against SARS-CoV-1 at 2.5 mM and SARS-CoV-2 at 10 mM, respectively [104,109]. The use of ACTs in malaria-endemic areas of Africa perhaps explains the later emergence and less serious impact of COVID-19 in those areas [111].

Treatment with artesunate-mefloquine (expected blood Cmax of 8.3 and 1 mM) led to replication inhibition above 70%. Additionally, artesunate exerted anti-inflammatory effects by decreasing the secretion of various proinflammatory cytokines [112]. The secretions of interleukin-1 beta (IL1beta), interleukin-6 (IL6), and interferon gamma were considerably increased due to cytokine storm [113,114]. In an in vitro inhibition of SARS-CoV-2 replication, Gendrot et al. showed that artesunate-mefloquine exerted high anti-SARS-CoV-2 activity with an inhibition of 72.1 ± 18.3%. In addition, other ACTs, including artesunate-pyronaridine, artesunate-amodiaquine, dihydroartemisinin-piperaquine, and artemether-lumefantrine, displayed the same range of inhibition (from 27.1 to 34.1%) [88]. These in vitro results reinforce the hypothesis that ACT drugs could be effective for anti-COVID-19 treatment [88]. An in vitro study against Vero E6 cells infected with a clinically isolated SARS-CoV-2 strain (IHUMI-3) of various antimalarial drugs showed low antiviral activity for dihydroartemisinin: EC_50_ 20.1 µmol/L, EC_90_ 41.9 µmol/L, CC_50_ 58.9 µmol/L, and SI 3) [115]. Molecular docking, along with in vitro studies of artemisinin-thymoquinone hybrids also demonstrated activity against the main protease of the virus [116].

In a phase II trial design study [117] to allow a rapid efficacy and toxicity assessment, camostat mesilate (serine protease inhibitor, 100 mg tablet, oral, two tablets, three times a day) and *A. annua* leaf tea (brewed tea from two 8 oz bags (225 mg per bag), three times a day (1350 mg/day)) were used immediately after COVID-19 positive testing. The hypothesis of this study was that the addition of agents that inhibit viral entry or replication of the SARS-CoV-2 virus will reduce the rate of a composite outcome of hospitalization due to COVID-19 pneumonia and will improve the condition by reducing the virus load [117].

## 8. *Artemisia* and Zinc

Zinc is as an essential micronutrient that is required to mount an effective antiviral response [118,119]. It is also critical in generating both innate and acquired (humoral) antiviral responses. The use of cellular zinc metalloproteases is effective for controlling virus entry and coronavirus fusion, and for increasing the intracellular Zn^2+^ concentration with zinc-ionophores which can efficiently impair the replication of a variety of RNA viruses, including SARS-CoV [120]. It has been reported that *A. annua* possesses a high concentration of zinc [75,106]. The flavonoids and other phenolic compounds present in *A. annua* also act as potent zinc ionophores [120,121]. Quercetin, one of the most abundant polyphenolics found in *A. annua*, plays a relevant beneficial role [77], in part, based on its antioxidant actions, which are partially derived from its interaction with iron, copper and zinc [118,119,120,121].

## 9. Brief Description of SARS-CoV-2 Genome and Possible Targets for Inhibition and Mode of Action

The genome of SARS-CoV-2 encodes several structural proteins such as spike (S) protein, membrane (M) protein, envelope (E) protein, and nucleocapsid (N) protein. The S protein functions as a major inducer of host immune responses and can interact with the host cluster of differentiation 147 (CD147) and angiotensin-converting enzyme 2 (ACE2) receptor, primed by trypsin-like proteases, cathepsins, and serine protease transmembrane protease serine 2 (TMPRSS2), and subsequent fusion of the human and viral cellular membranes, followed by viral invasion into the host cell [122,123]. The virus is internalized in a vesicle, whose protective capsid is then removed, allowing the genomic RNA to be liberated into the cytoplasm [124,125]. This is followed by proteolytic processing of replicase polyproteins, pp1a and pp1ab, by cysteine proteases, SARS-CoV-2 papain-like protease (PL^pro^), and SARS-CoV-2 main protease (M^pro^), also referred to as the 3-chymotrypsin-like protease (3CL^pro^) [126,127,128,129,130,131]. PL^pro^ and M^pro^ digest the first three cleavage sites and the remaining 11 sites, respectively, resulting in the release of the sixteen functional non-structural proteins (nsps). These nsps are essential for viral replication and transcription of the genome [132]. This is followed by virus assembly, and subsequently, virions are released from the infected cell through exocytosis to infect other cells and organs in the body.

Of interest, Wambier and Goren reported that androgens could upregulate the expressions of TMPRSS2 protein and ACE2 receptor [133]. Artemisinin can induce androgen receptor degradation and can disrupt the androgen response [134]; therefore, it might limit the expression of ACE2 and TMPRSS2 in sensitive cells, and thus inhibit SARS-CoV-2 infection [135]. CD147, a transmembrane glycoprotein, can increase the synthesis of matrix metalloproteinases (MMPs) and proinflammatory cytokines [136]. Artemisinin at 20–80 µg/mL inhibited the expression of CD147 [136], suggesting that it might also be effective [135].

Nrf2 signaling, a transcription factor, has been shown to reduce oxidative stress, and to attenuate pulmonary fibrosis by upregulating antioxidant expression and defence enzymes, and thus, contribute to disease progression [137,138,139]. It has been reported that *A. annua*, possessing potent antioxidant activity, and its constituents, such as artemisitene, can activate Nrf2 signaling that suppresses oxidative stress and inflammation [137,140]. Interestingly, artesunate has been shown to be a promising agent for improving lung fibrosis by inhibiting the activity of profibrotic molecules [135,141].

NF-κB is a protein complex that regulates cell survival, and stimulates proinflammatory cytokine production. An increase in cytokine production results in a cytokine storm (CS) which induces fatal inflammation [142,143]. Artesunate might inhibit NF-κB signaling to attenuate the cytokine storm, and thus, reduce the inflammatory response and lung inflammation [135,142].

Artesunate can inhibit the production of IL-1B, IL-6, and IL-8 by inhibiting NF-κB translocation in a dose-dependent manner in vitro [143]. Elevated IL-6 serum levels in COVID-19 patients may be a sign of cytokine release syndrome, suggesting that controlling IL-6 could decrease the natural course of the disease [144]. In addition, artemisinin/and or artesunate may limit CS by either inhibiting nuclear factor-κB (IκB) kinase (IKK), and thus over-active NF-κB signaling, or may inhibit the transcriptional activity [145,146].

Based on the aforementioned description, substances with a possible beneficial effect may act in various stages: (a) restricting internalization by either the binding of the virus to the receptors or inhibiting the function of the receptor itself, (b) inhibiting viral replication by blocking and/or inhibiting the activities of proteases, (c) helping the cell to resist viral attack, (d) blocking the spread of the virus, and (e) modulating the inflammation.

The targets that are currently being explored for the development of COVID-19 inhibitors include: S protein, ACE-2, TMPRSS2, and furin, as these are involved in the process of virus internalization; and viral proteases such as RdRp, PL^pro^, and M^pro^, as these are involved in virus transcription and replication [146,147,148,149]. Numerous studies are being pursued to identify potent inhibitors through the combination of computer-aided drug designing approaches and biochemical assays [5].

Of all the targets that are being explored for antiviral drug development, M^pro^ is one such structural protein emerging as a promising target due to is role in viral replication and transcription [150,151]. Structurally, Mpro is a dimer, each monomer of which consists of three domains, namely domains I, II, and III. The substrate-binding site containing the catalytic dyad (Cys145 and His61) is positioned between domains II and III [129]. In general, inhibitors first bind noncovalently with the enzyme such that the “warhead” is in close vicinity with the catalytic residue which is followed by a nucleophilic attack by Cys145 resulting in the formation of a covalent bond, thereby, inhibiting the enzyme either reversibly or irreversibly [152,153].

## 10. Inhibition Potential of *Artemisia* Constituents, including Artemisinin and Its Derivatives “Artemisinins” (such as Artesunate and Artmether) against SARS-CoV-2 Proteases

As noted earlier, artemisinin and some of its derivatives such as artesunate, artmether, and dihydroartemisinin, have exhibited broad-spectrum antiviral activities against pathogenic human viruses [154,155]. Notably, recent docking studies have indicated that artemisinin and artesunate could bind to the SARS-CoV-2 spike protein in a way that would interfere with its docking onto the human ACE2 receptor protein, which is the required first step in the host infection process of COVID-19 [156,157], and thus, restrict virus entry. The anti-SARS-CoV-2 activity has been attributed to inhibition of the spike protein mediated and TGF-β-dependent early steps in the infection process [158]. It is noteworthy that the incidence of COVID-19 and related deaths has been very low in countries with regular use of artemisinin-based antimalaria drugs [159]. Consequently, artemisinin has recently been repurposed as a potential COVID-19 drug [154]. Li et al., reported the results from an open-label nonrandomized study in which 41 COVID-19 patients received either standard of care (SOC) therapy (control) or SOC combined with artemisinin plus piperaquine (AP) [160]. Patients in the AP group showed faster recovery than control patients, reflecting the importance of artemisinin-based antimalarials for COVID prevention.

Screening by Sehailia and Chemat [161] of artemisinin and derived compounds reflected a better Vina docking score of −7.1 kcal mol^−1^ for artelinic acid. Artesunate, artemisinin, and dihydroartemisinin (artenimol) showed interactions with Lys353 and Lys31 of the spike protein receptor. A molecular dynamics analysis confirmed the stability of the formed complexes in the active site of their respective targets, thus, preventing infection [161].

In a recent study [162] to investigate the potential of artemisinin and its derivatives as possible inhibitors of SARS-CoV-2 nsp1, a key virulence factor suppressing the host’s immunological responses, various computational approaches reflected that artemisinin bound to nsp1 with a binding energy of −6.53 kcal/mol and with an inhibition constant of 16.43 mM. Three derivatives, i.e., artesunate, artemiside, and artemisone, showed binding energies of −7.92 kcal/mol, −7.46 kcal/mol, and −7.36 kcal/mol, respectively. Interactions (hydrophobic and hydrogen bonding) with Val10, Arg11, and Gln50 seemed to be responsible for the stabilization of the protein–ligand complexes. Accordingly, artemisinin and its derivatives may be promising for the development of drugs to inhibit SARS-CoV-2 nsp1 protein [162].

In silico molecular docking studies by Rolta et al. [163] to find the antiviral significance of phytocompounds showed that artemisinin had the best binding affinity with spike glycoprotein (PDB ID: 6VXX), spike ectodomain structure (PDB ID: 6VYB), and SARS coronavirus spike receptor-binding domain (PDB ID: 2AJF) with Etotal values of −10.5 KJ mol^−1^, −10.3 KJ mol^−1^, and −9.1 KJ mol^−1^, respectively. The study also revealed that artemisinin bound: (1) to spike glycoprotein (6VXX) via weak H-bonds with THR 778 and SER 730, and hydrophobic interactions with LEU 865, PHE 782, ASP 867, PRO 863, HIS 1058, ILE 870, ALA 1056, GLY 1059, and VAL 729; (2) to SARS-CoV-2 spike ectodomain structure (6VYB) via weak H-bonds with SER 730 and THR 778, and hydrophobic interactions with HIS 1058, ALA 1056, GLY 1059, VAL 729, PRO 863, LEU 865, PHE 782, ILE 870, and ASP 867; (3) to SARS coronavirus spike receptor-binding domain (2AJF) via hydrophobic interactions with PHE 390, ARG 393, ASP 350, and PHE 40 [162]. Thus, artemisinin can be effective in blocking the interaction of the SARS-CoV S protein with ACE2, thus, inhibiting its entry into the host cell.

In a blind molecular docking approach to identify possible main protease inhibitors, Das et al. screened 33 compounds, including artemisinin, and found that it interacted with M^pro^ (PDB: 6Y84) crucial binding sites, MET49, CYS145, and HIS163 (estimated free energy (ΔG) −7.15 kcal/mol and fullfitness score (kcal/mol) (FFS) of 1233.81 kcal/mol) [164]. Thirty-six phytochemicals from selected Arabic plants were tested as SARS-CoV-2 M^Pro^ inhibitors via an in silico molecular docking study with M^pro^ (PDB ID: 6LU7). The binding energies for artemisinin and artesunate were found to be −7.78 Kcal/mol and −6.46 Kcal/mol, respectively [165]. Targeting Mpro, the in silico computational relationship between sixty-two plant-derived natural drugs approved by the USFDA and the coronavirus main protease (PDB: 6LU7) protein suggested docking scores for artemisinin derivatives of: artenimol, −5.178 kcal/mol; artesunate, −4.862 kcal/mol; and artemether, −4.764 kcal/mol [166]. Sudeep et al. [167] investigated 25 natural compounds for their anti-host receptor glucose-regulated protein 78 (GRP78) and anti-SARS-CoV-2 M^pro^ activity via in silico molecular docking studies. The binding energy values of artemisinin with the GRP78 receptor and M^pro^ were determined as −7.89 and −8.06 kcal/mol, respectively [167].

The in silico probing results [168] showed that artemisinin and its derivatives (deoxyartemisinin, dihydroartemisinin acetate, artemisinic aldehyde, and deoxyartemisinin) manifested good oral absorption and bioavailability scores (0.55). These bound specifically to the Cys145 residue of M^pro^ via two to three hydrogen bonds with binding affinities ranging between −5.2 and −8.1 kcal/mol. Furthermore, artemisinin interactions with angiotensin converting enzyme 2 (ACE2) were dependent on the ACE2 allelic variants. A molecular dynamic simulation showed sufficient stability of the artemisinin–M^pro^ complex. These binding interactions, together with drug-likeness and pharmacokinetic findings, confirmed that artemisinin might inhibit Mpro activity and explained the ethnopharmacological use of the herb and its possible antiviral activity against SARS-CoV-2 infection inducing COVID-19 [168].

In a study by Patel et al. [169], SARS-CoV-2 M^pro^ (6LU7) was docked with bergenin, quercitrin, and dihydroartemisinin, and lower binding energy values as well as maximum interactions with active site residues of M^pro^ were evaluated for selecting the best pharmacophore-like drug candidates. Dihydroartemisinin had the lowest binding energy, with a value of −7.23 kcal/mol and formed hydrogen bonds, electrostatic interactions, and hydrophobic interactions with THR190, GLU166, GLN189, GLY143, HIS163, HIS164, CYS145, and PHE140. These results suggest that dihydroartemisinin may be a potent M^pro^ inhibitor [169].

Sharma and Deep investigated FDA-approved drugs and natural compounds for targeting M^pro^ and compared docking and MD simulation results of complexes of drugs with those of of inhibitor N3 (experimentally obtained). Artesunate was found to be one of the potent compounds for binding (binding energy of −8 kcal/mol) [170]. Drugs and bioactive compounds (having antimalarial, antiviral, anti-inflammatory, and HIV protease inhibiting activities) were tested against the SARS-CoV-2 spike glycoprotein utilizing molecular methodologies (molecular docking, virtual screening, and drug-like and ADMET prediction) to identify inhibitors [171]. Based on docking scores, H-bonds, and amino acid interactions, artemisinin (binding energy, −6.8 kcal/mol; H-bonds, 2; KI, 15.37 µmol/L) was reported to show a poor affinity for S protein [171].

Roy Chattopadhyay [172] performed in silico analyses on some FDA-approved drugs to study the mechanism of SARS-CoV-2 infection and the interactions of various drugs with its proteins, such as RdRp, helicase protein, nucleocapsid protein (NC), S protein RBD, envelope protein (E), nsp10, nsp14, and nsp15. In this study, drugs with at least one viral protein interaction exhibiting a minimum binding energy of −0.7 kcal/mol were considered to be appropriate. Artesunate exhibited binding to proteins: E protein, −7.2 kcal/mol; helicase protein, −7.1 kcal/mol; nsp10, −7.6 kcal/mol; nsp14, −8.4 kcal/mol; nsp15, −8.2 kcal/mol; and NC protein, −8.8 kcal/mol. Artemether’s binding to proteins was: helicase protein, −7.5 kcal/mol; nsp10, −7.0 kcal/mol; nsp15, −7.4 kcal/mol; and NC, −8.0 kcal/mol. Thus, artesunate and artemether can act in several ways as SARS-CoV-inhibitors [172].

Using virtual screening, molecular docking, toxicity analysis, and MD simulations (docking stability), with HCQ as a positive control, 203,458 natural compounds were screened for inhibition of the ACE-2–S protein complex. Artemisinin was found to be one of the four final compounds, along with andrographolide, pterostilbene, and resveratrol. Artemisinin and andrographolide were the least toxic, and the binding score for artemisinin was −6.2 kcal/mol [173].

Various antiviral drugs were screened for inhibition of nsp15 [174]. In an in silico study, binding affinity, estimated KI, orientation of molecules in the active sites, and key interactions with residues of nsp15 were utilized to identify candidates, among which artesunate was one of the most promising, along with simeprevir and paritaprevir. The binding energy of artesunate was −7.2 kcal/mol and the estimated KI 5.275 was µmol/L. The artesunate–nsp15 residue interactions were with LYS290, SER294, THR341, and TYR343 (hydrogen bonds); HIS250, HIS235, and TRP33 (π interactions); and GLY247, GLY248, VAL292, CYS293, GLU340, and LYS345 (van der Waals interactions) [174].

A library of several anti-inflammatory and antiparasitic drugs was screened [175] to access the binding affinity with 3CL^pro^, PL^pro^, RdRp, S protein, helicase protein, nsp1, nsp3, nsp4, nsp9, and nsp16–nsp10. Artesunate, in an in silico molecular docking study based on the results of drug–protein complexes, exhibited significant binding (docking score −8.1 kcal/mol) with nsp3. Artesunate formed hydrogen bonds with ALA154, PHE156, ASP157, and LEU126, along with alkyl and π-alkyl interactions with VAL49, ILE23, ALA52, and PHE156, which increased its binding stability with nsp3 [175].

Secondary metabolites of Ayurvedic medicines were screened for their potential inhibition of SARS-CoV-2 proteins: 3CL^pro^ (nsp5), PL^pro^ (nsp3), RdRp, helicase (Hel) protein, S protein, M protein, NC protein, E protein, hACE-2 receptor, nsp1, nsp2, nsp4, nsp6, nsp7-nsp8, nsp9, and nsp10-nsp16. In silico molecular docking and MD simulation studies suggested that artemisinin exhibited inhibition efficacy scores of −5.174 kcal/mol; and −6.134 kcal/mol for binding with nsp2 and PL^pro^, respectively. Artemisinin formed only one H-bond with ASP108 of PL^pro^ [176].

In a study by Ribaudo et al. [177], computational techniques were adopted, including docking, to study the structural details and stability of the artemisinin/dihydroartemisinin–S protein RBD–ligand complexes. The complexed protein backbones reached stabilization within less than 5 ns of simulation time. RMSD values (average ± standard deviation) of 2.51 ± 0.24 Å and 2.15 ± 0.18 Å were measured for the backbones of RBD–artemisinin and RBD–dihydroartemisinin complexes, respectively. The binding of artemisinin and dihydroartemisinin was also investigated using bio-layer interferometry. Dihydroartemisinin showed weaker binding and worse correlation (KD = 66.5 µM, R^2^ = 0.5210) than artemisinin (KD = 51.4 µM, R^2^ = 0.6264). The results of this study support the hypothesis that “artemisinin” may act through a combination of mechanisms when exploiting its antiviral function and RBD could be one of the macromolecular targets [177].

Among 13 antimalarials tested, and with remdesivir as the control, docking studies [178] revealed that artemether exhibited interactions with the SARS-CoV-2–ACE2 complex (6M0J), with a GScore of −7.09. On docking with SARS-COV-2 M^Pro^ (6LU7), artemether showed binding with a GScore value of −4.09. Thus, the in silico approach suggested that artemether may be effective for repurposing [178]. Dey et al. [179] used a combination of molecular docking, all-atom molecular dynamics simulation, and MM-PBSA analysis to test four drugs—Tretinoin, Mefenamic Acid, Ondansetron and Artemether—as potential inhibitors of ion channels formed by the SARS-CoV-2 E protein. Artemether showed interactions with PHE4 (Chains A–E) only and the binding affinity calculation of the docked complexes showed that it possessed the lowest binding affinity of −7.0 kcal/mol. Thus, artemether can be a SARS-CoV-2 E protein ion channel blocker and virus assembly inhibitor [179].

Rai et al. [180] performed an in silico investigation of the binding of some components of *A. annua*, including flavonoids, phenolics, and terpenoids, with protease ORF1a and found that artemisinin and β-artether interacted strongly with GLY, SER, and LEU (binding scores of −176.24 and −212.11, respectively) in a manner quite similar to the interactions observed for remdesivir, hydroxychloroquine, and ivermectin. The docking results of artemisinin and artesunate with RdRp showed interactions with conserved core amino acid (ASN, LYS, TYR, and PHE) residues. Artemisinin also exhibited interactions with helicase receptor and ACE-2 receptor. Based on these docking studies, Rai et al. concluded that artemisinin, β-artether, artesunate, and eupatorin have strong binding energies, docking scores, and close interaction with core amino acid residues equivalent to remdesvir and ivermectin against SARS-nCOV [180].

Tang et al. [181] employed molecular docking and network analysis to elucidate active components or targets and the underlying mechanisms of *A. annua* for the treatment of COVID-19. Through molecular docking simulation and computing binding free energy, three flavonoids, namely quercetin, isorhamnetin, and kaempferol, and particularly quercetin and isorhamnetin, showed excellent binding affinity with seven hub targets. An in vivo study showed that isorhamnetin could inhibit the SARS-CoV-2 spike pseudotyped virus from entering ACE2h cells [182]. The MD and MM-GBSA calculation data further indicated that MPK1/quercetin and TP53/kaempferol possessed the highest binding free energy, which demonstrated the repurposing possibilities of quercetin and kaempferol based on their binding activity with multiple COVID-19 targets [181].

The potency of artemisinin and its six derivatives, i.e., artemether, arteether, artesunate, dihydroartemisinic acid, dihydroartemisinin, and artemisinic acid, has been evaluated against M^pro^ by molecular docking studies [183]. These studies have indicated that all ligands have similar interactions in the active pocket of M^pro^, with good binding affinity. However, artesunate was located in the active region of the protein more strongly (making four H-bonds through carbonyl groups of the ligand and NH moiety of GLY143, SER144, CYS145, and GLU166 polar residues with bond distances of 2.18, 2.95, 2.16, and 1.93 Å, respectively) than the other artemisinin derivatives, with a docking score of −9.35 kcal/mol. The carbonyl moiety of the GLN189 residue also makes water-bridged hydrogen bonding interactions with the oxygen atom of artesunate, with a bond distance of 1.78 Å. Hydrophobic interactions were also established between the THR25 and HIS41 residues and the endoperoxide bridge moiety of artesunate. Dihydroartemisinic acid and dihydroartemisinin, with docking scores of −8.49 and −8.41 kcal/mol, had the closest score to artesunate. Artemisinin exhibited H-bond interactions with ASN142, GLY143, SER144, and CYS145, and hydrophobic interactions with HIS41 and HIS163, whereas other artemisinin derivatives also showed similar interactions, especially with THR25, ASN142, GLY143, SER144, CYS145, HIS41, MET165, GLU166, and GLN189 residues. Thus, artesunate, dihydroartemisinic acid and dihydroartemisinin, with binding energies between −8.42 and −9.35 kcal/mol, had promising results for M^pro^ inhibition [183].

The in vitro anti-SARS-CoV-2 potential of nine artemisinin-related compounds has been investigated by Cao et al., who carried out a time-of-drug-addition assay [158]. Arteannuin B showed the highest anti-SARS-CoV-2 potential with an EC_50_ of 10.28 ± 1.12 µM; artesunate and dihydroartemisinin showed similar EC_50_ values of 12.98 ± 5.30 μM and 13.31 ± 1.24 μM, respectively. Mode of action analysis revealed that arteannuin B and lumefantrine acted at the post-entry step of SARS-CoV-2 infection. These studies also suggested that artesunate could inhibit SARS-CoV-2 replication in a dose-dependent manner. Combined with the safety and potential immunoregulatory activities of artemisinins, Cao et al. concluded that these might represent a potential medical countermeasure against COVID-19 [158].

A recent study by You et al., demonstrated that dihydroartemisinin exerted therapeutic effects against bleomycin-induced pulmonary inflammation and secondary pulmonary fibrosis (PF) by inhibiting activated Janus kinase 2 (JAK2), a signal transducer and activator of transcription 3 (STAT3) expression. It also inhibited alveolar inflammation, and attenuated lung injury and fibrosis, possibly representing its importance to treat PF associated with COVID-19 [184].

It has also been shown that artesunate was more potent than the *A. annua* plant extracts, artemisinin and artemether (the last two were found not to be effective against the virus) with EC_50_ values of 7 μg/mL (3.4 μM), 128–260 μg/mL (7.3 μM), 151 μg/mL (535 μM), and >179 μg/mL (>600 μM), respectively, on Vero E6 cells, and with similar results on human hepatoma Huh 7.5 cells. It is notable that almost complete inhibition of viral replication was obtained for 15 μg/mL and 22 μg/mL on Vero E6 and Huh 7.5 cells, respectively [12,91].

In a recent study [185], several artemisinin- and quinoline-based hybrid compounds were synthesized and analyzed in vitro for their SARS-CoV-2 inhibitory activity in a cytopathic effect reduction assay. All artesunic acid-containing hybrids displayed superior potency against SARS-CoV-2 (EC_50_ values 7.8–46 μM) and showed either low or no cytotoxic effects on Vero E6 cells (CC_50_ up to 110 µM). The most active artesunic acid-derived hybrid was significantly more potent in vitro (EC_50_ = 7.8 µM) than its parent compound, artesunic acid (EC_50_ > 50 µM). Among the quinoline-based new compounds, quinoline-adamantane (EC_50_ = 1.5 μM) was the most efficient in vitro, outperforming the reference drugs chloroquine (EC_50_ = 3.8 µM) and remdesivir (EC_50_ = 4.0 µM) [180]. The use of quinoline and artemisinin classes of antimalarial drugs effective against SARS-CoV-2 in vitro and in vivo, in clinical settings, has been reviewed by Firestone et al. [186].

In a prospective study [187], 43 cases of confirmed COVID-19 patients were divided into routine treatment (*n* = 25) and artesunate treatment groups (*n* = 18). The routine treatment group received lopinavir/ritonavir, 500 mg + α-aerosolized interferon 500 × 104 U, twice daily; the artesunate treatment group was given artesunate, 60 mg twice daily, in addition to the routine treatment for 10 days. In the artesunate treatment group, the time for significant improvement of symptoms (days: 3.33 ± 1.91 vs. 4.84 ± 2.19), negative conversion time of COVID-19 nucleic acid (days: 4.72 ± 2.16 vs. 6.68 ± 3.76), lung lesion absorption starting time (days: 5.39 ± 2.36 vs. 7.48 ± 3.78), lung lesion absorption greater than 70% time (days: 14.11 ± 4.16 vs. 17.04 ± 4.42), and the length of hospital stay (days: 16.56 ± 3.71 vs. 18.04 ± 3.97) were significantly shorter than those in the routine treatment group. Thus, artesunate shortened the treatment time for COVID-19 [187]. From the experience of treatment of severe falciparum malaria, it is conceivable that, for the treatment of COVID-19, it is best to start with a high initial IV dose of artesunate, i.e., 4–8 mg/kg/b.w or 280–560 mg for a 70 kg person, given as an IV bolus infusion at 10–12 h intervals to achieve ≥10 µM serum concentration or 300–3000 ng/mL or even higher for the first exposure. For the best results and to prevent progression of the disease, treatment should be a short course therapy of ≥3 days, which will cover ≥7 replication cycles of COVID-19 at the early stages of symptomatic disease, which is associated with robust viral replication. Thus, artesunate may be a potential agent for the treatment of moderate to severe COVID-19 infection [187,188].

In vitro studies have shown that ACTs containing pyronaridine-artesunate (in a 3:1 ratio) were significantly effective in the human lung epithelial cell line Calu-3 [189]. Pyronaridine has demonstrated in vitro antiviral effects on SARS-CoV-2 in a human lung epithelial cell line, while artesunate, in addition to antiviral effects, has shown anti-inflammatory properties via IL-6-mediated pathways, reflecting possible benefits for COVID-19 treatment [172]. Another ACT, mefloquine-artesunate, has also shown potent antiviral activity with increased drug concentration in lung tissue, a potential clinical advantage in COVID-19. The safety of ACTs has been established in children and adults with malaria, providing some reassurance for their use in COVID-19 treatment [190].

Herb ingredient–target function action networks have been utilized to elucidate the potential mechanisms of Traditional Chinese medicine (TCM) herbs and in this relationship network, *A. annua* was identified as one of the eight commonly used herbs, and artemisinin as one of the twelve main ingredients, targeting viral protein and other key targets and reducing viral infection and inflammatory storm [191]. The established immune-modulatory properties and potential involvement of autophagy of artesunate have also been considered to be responsible for the beneficial effects in critically ill patients with COVID-19 [192].

Artemether, artesunate and, arteannuin B remarkably reduced pangolin coronavirus GX_P2V infection (artemether (EC_50_ = 3.701 µM, CC_50_ > 200 µM, SI > 54.04), artesunate (EC_50_ = 10.10 µM, CC_50_ = 127.3 µM, SI = 12.60), and arteannuin B (EC_50_ = 8.838 µM, CC_50_ = 116.9 µM, SI = 13.23)) [193]. The time-of-addition assay and Western blot showed that artemether functioned at both entry and post-entry stages, whereas the other two compounds functioned at the post-entry stage. When artemether was added at 6.25 µM, the expression of SARS-CoV-2 (isolate WIV04, accession No. MN996528.1) NP protein was almost completely inhibited. Twenty-five µM arteannuin B and 25 µM artesunate also achieved the same inhibitory effect for viral NP proteins. Artesunate (EC_50_ = 16.24 µM, CC_50_ = 127.3 µM, SI = 7.84) and arteannuin B (EC_50_ = 12.03 µM, CC_50_ = 116.9 µM, SI = 9.72), showed potent anti-SARS-CoV-2 virus activity. These findings suggest that artemether, artesunate, and arteannuin B have potential for the inhibition of SARS-CoV-2 in vitro [193].

## 11. Concluding Remarks

In summary, extensive in vitro and in vivo data have revealed that *A. annua*, artemisinin, arteannuin B, and/or its derived products “artemisinins” (dihydroartemisinin, artemether, artesunate, etc.) have a broad spectrum of biological abilities (including antiparastic, antifungal, antibacterial, anti-inflammatory, immunoregulatory, anticancer, and antiasthmatic) and antiviral properties. The anti-COVID-19 effects and mechanisms of *Artemisia* and its constituents include, but are not limited to: (1) inhibiting SARS-CoV-2 invasion and replication by targeting the key proteins of spike, ACE2, spike–ACE2 interaction, TMPRSS2, and NSPS, including M^pro^, PL^pro^, and RdRp; (2) regulating immune and inflammatory responses by targeting inflammatory cytokines and chemokines; (3) protecting against ARDS and MODS by suppressing the crosstalk of viral toxicity, endothelial damage, and cytokine storm. Artemisinin and its derivatives are already known for their powerful bioactivity, tolerability, and relative affordability. The in vitro findings have led researchers to suggest that one or more compounds in *A. annua,* either not yet identified or acting in synergism, may point to a safe, low-cost therapeutic treatment for SARS-CoV-2, the virus responsible for the COVID-19 pandemic. Thus, *Artemisia*-based formulations may be either new, safe and cost-effective therapies or even be used as antiviral nutraceuticals in boosting immunity and providing tolerance to virus infections. However, further studies need to be undertaken to determine in vivo efficacy.

## Figures and Tables

**Figure 1:** Chemical structure of artemisinin (**1**), dihydroartemisinin (**2**), artemether (**3**), artesunate (**4**), and arteannuanin B (**5**).

## Data Availability

The data presented in this study are available on request from the corresponding author.
